# PSR: Unified Framework of Parameter-Learning-Based MR Image Superresolution

**DOI:** 10.1155/2021/5591660

**Published:** 2021-04-21

**Authors:** Huanyu Liu, Jiaqi Liu, Junbao Li, Jeng-Shyang Pan, Xiaqiong Yu

**Affiliations:** ^1^School of Electronics and Information Engineering, Harbin Institute of Technology, Harbin 150001, China; ^2^Center of AI Perception, AI Research Institute, Harbin Institute of Technology, Harbin 150001, China; ^3^College of Computer Science and Engineering, Shandong University of Science and Technology, Qingdao 266590, China; ^4^32021 Troops of the PLA, Beijing 100094, China

## Abstract

Magnetic resonance imaging has significant applications for disease diagnosis. Due to the particularity of its imaging mechanism, hardware imaging suffers from resolution and reaches its limit, and higher radiation intensity and longer radiation time will cause damage to the human body. The problem is expected to be solved by a superresolution algorithm, especially the image superresolution based on sparse reconstruction has good performance. Dictionary generation is a key issue that affects the performance of superresolution algorithms, and dictionary performance is affected by dictionary construction parameters: balance parameters, dictionary size, overlapping block size, and a number of training sample blocks. In response to this problem, we propose an optimal dictionary construction parameter search method through the experiment to find the optimal dictionary construction parameters on the MR image and compare them with the dictionary obtained by multiple sets of random dictionary construction parameters. The dictionary we searched for the optimal parameters of the dictionary construction training has more powerful feature expressions, which can improve the superresolution effect of MR images.

## 1. Introduction

Magnetic resonance imaging (MRI) becomes more and more widely used in medical clinical applications and plays an increasingly important role in the diagnosis of various diseases [1–5]. The mechanism of MR imaging is different from that of natural images. The hydrogen protons of human organs are magnetized under the action of external magnetic fields and generate a magnetic resonance phenomenon under the action of a magnetic field. The changing magnetic signals are converted into electrical signals by induction coils and fill the *K* space. Finally, an MR image is generated through the Fourier transform. The method of improving resolution relies heavily on increasing the magnetization of more free water in human tissues and organs [6], which will cause the increase of the radiation time and radiation intensity of the main magnetic field of the magnetic resonance imager and the loaded electromagnetic waves [7]; excessive radiation can lead to serious consequences, such as overheating of the human body and protein inactivation [8], causing harm to the human body and not suitable for clinical application. From the perspective of current imaging methods and technologies, the hardware imaging resolution reaches the limit value. To increase the resolution, software superresolution technology must be used to increase the image resolution.

Image superresolution methods are mainly based on interpolation, reconstruction, and learning. Li and Orchard [9] proposed a new edge-directed image interpolation (NEDI) method; Wang and Ling [10] proposed an Edge-Adaptive Interpolation Algorithm (EAIA), combined with bilinear and NEDI methods; Giachetti and Asuni [11] proposed an interpolation based on iterative curvature method based on the NEDI method. But the interpolation-based method does not essentially increase the image information. Irani and Peleg [12] proposed an iterative backprojection method (IBP), Schultz and Stevenson [13] proposed a superresolution method based on maximum posterior probability (MAP), Patti et al. [14] proposed the convex set projection method, *and* in [15], the projection onto convex sets superresolution reconstruction method was used for the superresolution of cardiac valve MR images. POCS algorithm is not good at maintaining the image edge and can not restore the high-frequency information on the image. The superresolution method based on reconstruction regards low-resolution observation images as a constraint condition of the original high-resolution image, and a series of solution spaces satisfying the constraint condition can be obtained through the alternating iteration method. Most of the above algorithms use prior knowledge such as the edge characteristics of the image, the nonnegativity of pixels and local smoothing characteristics to construct constraints and then solve the optimization problem through an iterative algorithm. The reconstruction algorithms are computationally expensive, and the resulting image is reconstructed too smoothly. Learning-based superresolution methods mainly include dictionary learning and deep learning. Yang et al. [16] proposed a superresolution reconstruction algorithm based on sparse representation. This method effectively overcomes the problem of inaccurate representation caused by using a fixed number of neighbors. On the basis of the methods [17], adaptive sparse field selection and adaptive regularization are applied to superresolution. Yang et al. [18] proposed a double-geometric neighborhood embedding method (DGNE), which uses multiview features and local spatial neighbors of image blocks to find image features-spatial manifold embedding. Zhang et al. [19] combined subspace division and local regressor learning through the mixture of experts method to further improve the quality of image reconstruction. With the development of deep learning. Shi et al. [20] propose a novel image SR method that integrates both locals and global information for effective image recovery. This is achieved by, in addition to TV, low-rank regularization that enables utilization of information throughout the image. The reconstructed image will produce stripe distortion, and the texture and other details will be blurred to some extent. Dong et al. [21] used convolutional neural networks for image superresolution reconstruction for the first time. This method first uses bicubic interpolation to enlarge it to the target size and then passes through a three-layer convolution network doing the nonlinear mapping. The results obtained are output as high-resolution images, and experiments show that it has achieved good results. Since then, Residual Dense Network [22], SRGAN [23], and many deep networks [24, 25] are proposed and used. Deep learning methods are based on data driving, and Network performance is affected by the amount of data. However, due to the particularity and privacy of MR images, it is difficult to obtain large amounts of data. MR image superresolution task is more suitable for methods that weak dependence on data volume.

Our contributions are threefold. First, we propose a superresolution architecture based on joint dictionary learning suitable for a small number of MR images. Second, we analyze the effect of dictionary parameters on dictionary performance and find the optimal dictionary parameters through parameters learning. Third, experiments prove that our proposed method can achieve state-of-the-art performance, even if there are only a few image data.

## 2. Algorithm and Analysis

### 2.1. Algorithm

We propose a superresolution architecture based on joint dictionary learning suitable for a small number of MR images. The algorithm framework is shown in Figure 1. Through corresponding high and low-resolution image block training, learn high and low-resolution dictionary, low-resolution image blocks are sparsely represented by a low-resolution dictionary, and the sparse coefficients can be used for high-resolution image reconstruction. The performance of high and low-resolution dictionaries directly affects the image reconstruction effect.

Training a joint dictionary requires the use of high-resolution image block sets and low-resolution image block sets. Training image pair is represented by *P*={*Y*^*l*^, *X*^*h*^}. *X*^*h*^={*x*_1_, *x*_2_, *x*_3_,…, *x*_*n*_} and *Y*^*l*^={*y*_1_, *y*_2_, *y*_3_,…, *y*_*n*_} represents features extracted from image blocks. The dictionary training of two image feature spaces is expressed as follows [16]:

(1) $$\begin{array}{c} D_{h}=\arg\underset{\left\{D_{h},z\right\}}{\min}{\left\|X^{h}-D_{h}Z\right\|}_{2}^{2}+\lambda {\left\|Z\right\|}_{1}, \end{array}$$

(2) $$\begin{array}{c} D_{l}=\arg\underset{\left\{D_{l},z\right\}}{\min}{\left\|Y^{l}-D_{l}Z\right\|}_{2}^{2}+\lambda {\left\|Z\right\|}_{1}. \end{array}$$

According to the idea of the joint training method, the image blocks corresponding to the two image feature block spaces are concatenated to form a new image feature block space, so formula (3) [16] can be obtained:

(3) $$\begin{array}{c} \underset{\left\{D_{h},D_{l},Z\right\}}{\min}\frac{1}{N}{\left\|X^{h}-D_{h}Z\right\|}_{2}^{2}+\frac{1}{M}{\left\|Y^{l}-D_{l}Z\right\|}_{2}^{2}+\lambda \left(\frac{1}{N}+\frac{1}{M}\right)\times {\left\|Z\right\|}_{1}, \end{array}$$

*M* is the dimensions of the low-dimensional image feature block, and *N* is the dimensions of the high-dimensional image feature block. It can be seen from formula (3) that balance parameters, dictionary block size, overlapping block size, and the number of dictionary blocks have an important impact on the performance of the dictionary. We obtain the optimal parameters of dictionary construction through experimental analysis so as to achieve the improvement of dictionary performance and image reconstruction effect.

### 2.2. Parameter Set and Analysis

The parameter set is written as parameter = [*λ*, overlap, *n*, spn], where *λ* is balance parameter, the overlap is the size of the overlap block, *n* is the size of the dictionary block, and spn is the number of the exemplar patch.

From the mechanism of reconstruction perspective, changes of the parameter can cause changes in the structure and quantity of the data calculated by the dictionary, which has a great influence on the effect of reconstruction. The specific analysis is as follows.

According to the formula in equation (3), the balance parameter *λ* is used to balance sparsity and low-resolution dictionary sparse, which represents image block errors. It can be analyzed from the equation that the sparsity is inversely proportional to the error. In order to find the minimum sparsity coefficient, the error will increase, and vice versa, so there must be an optimal value *λ* to minimize the value of equation (3).

The overlapped block overlap is the size of the overlapped portion among the image blocks, and is divided into the selection of sample blocks in dictionary training and overlap of test image blocks in reconstruction. In order to ensure that the detailed features of the sample block can be extracted in the dictionary training, the maximum overlapped block method is used to select samples, which makes 1 pixel gradually change between the training sample blocks of a localized image. In order to eliminate the boundary blur caused by the feature extraction of the test image block and the reliability of the connection between the reconstructed blocks, the overlap between the blocks is required. The larger the overlap block, the larger the constraint between the reconstructed blocks, and the better the reconstruction effect.

MR images are expected to show various tissue structures clearly, with high tissue resolution. However, the outline of the diseased tissue can not be seen clearly and separated from the surrounding structure, so it is important to clearly display the texture details, especially the boundaries between different organizational structures, and to some extent, reduce the chances of misjudgment of the diagnosis due to the blurring of the picture. Then, for the dictionary and the reconstructed image, the size of the dictionary block used to represent the feature will affect the number of effective features. The smaller the dictionary block, the fewer features are generated, which makes the reconstructed image have limitations and larger errors, such as the most extreme 1 × 1 and 2 × 2 blocks. The features they can describe are limited. However, the oversized block is also problematic. The image is too large, and the features described by the image block can be combined and described by several smaller feature blocks, then they lose the properties of the feature block, such as extreme cases; the test image itself is a large feature block; of course, this is unreasonable. Therefore, there must be an optimal value for image segmentation, which makes image reconstruction better.

We adopt the method of sparse representation and reconstruction of image blocks. When training the dictionary, a large number of sampling image blocks are required. The number of image sampling blocks has a certain influence on the reconstructed quality. If the image block sample is too little, it is not enough to complete the training of the dictionary. If there are too many image sample blocks, especially the features of some image sample blocks that are not obvious or typical, the characterization of the dictionary cannot be improved even if there is much training. Is there an optimal number of partitions? Since the selected image sampling blocks are randomly extracted, it is difficult to extract the required sample blocks in an accurate number of blocks, so there is no optimal number of sample blocks. Therefore, the selection of the sample block is as long as a certain amount. Too little or too much can both not change the image reconstruction effect.

## 3. Experimental Results and Analysis

### 3.1. Dataset

The experiments are all set as follows: The method adopts the experimental framework of Section 1 of Chapter 2. 81; representative pictures of different categories in the image library were selected as the training samples of the high-resolution dictionary. These MR images were obtained from Siemens 3T platforms using a 32-channel head coil. Low-resolution images are generated by the degradation of high-resolution images. LR images are generated following the steps: (1) the high-resolution images are transformed from image space to *K* space by FFT, (2) in the *K* space, the outer high frequency is truncated, (3) through the inverse Fourier transform, the truncated *k* space data are transformed into the image space to generate the corresponding low-resolution images. This mimics the actual acquisition of LR and HR images by MRI scanners. In the experiment, as shown in Figure 2, five images corresponding to different types of MR images are selected as test samples.

### 3.2. Joint Optimization of Parameter

#### 3.2.1. Balance Parameter *λ*

The optimal value of the balance parameter is verified by the experiments below. The initial parameter configures are as follows: the dictionary size is 512, the balance parameter *λ* = 0.1, and the block size is 5 × 5, the overlap block is 4, the number of sample blocks is 100000, and the test samples are, respectively, selected from the head, ankle, carotid artery, knee, and neck, as shown in Figure 2.

It can be seen from Figure 4 that the value of PSNR decreases significantly with the increasing *λ* when *λ* > 0.1. On the contrary, when *λ* < 0.1, the value of PSNR decreases slowly with *λ* decreasing. As the balance parameter of the sparsity, *λ* exists optimal value, which makes PSNR maximum. For further verification, let *λ* = 0.1 as the optimal balance parameter. The super resolution ratio is 1 : 4.

The experiment used a superresolution ratio of 1 : 4, and other experimental parameters are the same as those in experiment ratio 1 : 2. The experimental results are shown in Table 2.

Figure 3 is obtained from Table 2. It can be seen from the figure that the extreme point is near *λ*=0.1, and the experiment with a superresolution ratio of 1 : 4 has the same conclusion as the experiment with a superresolution ratio of 1 : 2.

#### 3.2.2. Overlap Block

The relationship between the image reconstruction effect and overlapped blocks is verified by the following experiment. The initial parameters in the experiment are the same as those in Experiment Balance parameter, and the changed parameters are the size of the overlapped region. The overlapped blocks 1–4 are used to represent the superposed pixels. The experimental results can be seen in Table 3.

According to the experimental results, the images with superresolution ratios of 1 : 2 and 1 : 4 are demonstrated, respectively, in Figure 5, where the abscissa represents the number of overlapped blocks, and the ordinate is the corresponding PSNR. It can be seen from the figure that as the overlay area of the overlapped blocks decreases, the value of PSNR decreases. This is because the larger the overlay area where the image blocks selected for the reconstructed block, the larger the constraint between the reconstructed blocks, and this is easy to find the closest image block to be connected. The more the pixel points at the edge of the image block overlap, the easier it is to eliminate the truncation error caused by the feature extraction. It also has a certain inhibitory effect on noise.

#### 3.2.3. Dictionary Blocking Size

The following experiments show the quality of the reconstructed image when having the different blocking conditions for the same test image, where the set of dictionaries is generated with the altering size of the blocked image.

Other experimental parameters do not change, and the changed parameters are the block size of the image blocking. The image blocking of the dictionary has the same requirements as the image blocking of the test image.

The experimental results are as follows: when the superresolution ratio is 1 : 2, 8 high-definition dictionaries with the image block from 3 × 3 to 10 × 10 are generated. Three image blocks are shown in Figure 6. It can be seen that as the image block size increases, the dictionary block becomes more and more complicated. The resulting PSNR values are shown in Table 4.

Table 4 shows the value of the superresolution reconstruction PSNR corresponding to the different block training dictionaries of images. Since the reconstructed overlapped block is 4, which exceeds the block size of the sample block itself, the reconstructed samples are not correct when the dictionaries are, respectively, corresponding to block 3 × 3 and block 4 × 4. The two data sets are not analyzed. The other data corresponding to dictionary block and PSNR are shown in Figure 7.

The abscissa in Figure 7 only represents the block of the dictionary and the image. For example, the abscissa 5 indicates that the dictionary block is 5 × 5 and so on. Increasing the block size will reduce the value of PSNR when the overlap block size is unchanged. That is to say, the block is not bigger always better. When the block is large, the number of dictionary blocks that represent the image feature block will increase, and the reconstruction error will become larger. It can be seen that the preferred block value is 5 × 5 or 6 × 6 blocks, and the calculation efficiency 5 × 5 blocks is optimal.

When the superresolution ratio is 1 : 4, high-resolution dictionaries from 5 × 5 to 13 × 13 are generated through experiment. Three high-resolution dictionaries are shown in Figure 8, where the dictionary block becomes more and more complicated with the number of the blocks increasing. But the too-large block causes too many singular matrices when calculating the dictionary block, which causes the dictionary block information to be lost. The larger the block, the fewer the valid dictionary blocks. This will lead to a decrease in PSNR values, as shown in Figure 8(c). The parameters in the experiment only change is the superresolution ratio of 1 : 4, and the experimental results are shown in Table 5.

The data in Table 5 are the corresponding PSNR values generated by the superresolution reconstruction of the test sample with different block training dictionaries for the corresponding image. In order to intuitively distinguish the influence of the block on the reconstruction, the horizontal coordinate is the image block and the ordinate is the PSNR, as shown in Figure 9.

The abscissa in Figure 9 only shows the image blocking situation. The preferred PSNR corresponds to a 10 × 10 or 11 × 11 image blocking. Taking into account the calculation amount, 10 × 10 image blocking is the best. If the image blocking is too small, it cannot represent features fully, and if the image blocking is too large, the algorithm itself has limitations.

Comparing results corresponding to the superresolution ratios of 1 : 4 and 1 : 2, they have their own best partitions. The image blocks with a superresolution ratio of 1 : 4 are approximately double that of 1 : 2. This is because the image local information required for 4 times superresolution becomes larger, and naturally, the image block needs to be correspondingly larger.

The above two experiments compared the results where the overlapped blocks are fixed as 4. But in the overlapped block experiment, the larger the overlapped blocks, the better the results. The experiment did not consider the best case of overlapped blocks. Next, we will consider that if the best block changes when blocking the different overlapped blocks corresponding maximum.

The experiment verified the effect of the maximum overlap block experiment on the superresolution performance. The parameters are the same as those before the experiments. The changed parameters are only the block size and the overlapped block. For example, the block size is *n* × *n*, and the overlapped block value is *n* − 1. When the superresolution ratio is 1 : 2, the experimental results can be seen in Table 6.

The data show the superresolution reconstruction, where each test sample corresponds to different blocks and overlap blocks. For comparison, the data are plotted as shown in Figure 10.

The horizontal coordinate in Figure 11 only indicates the difference of the block. It can be clearly seen that the reconstructed effect is better from Figure 11 when the dictionary block is 5 × 5 or 6 × 6 blocks. The smaller blocks make the features of the blocks insufficient, and the too-large blocks need to increase the number of calculated pixels. The increase in the size of the dictionary representation block caused by the increase of the feature block makes the error larger and impacts the PSNR effect. In this experiment, the largest overlap block is used to make each component block reach the best reconstruction. It can be seen that the better block value is still 5 × 5 or 6 × 6, and it is best to select a 5 × 5 block for the calculation efficiency.

The above experiment verified the effect of the maximum overlap block experiment on the superresolution performance. The parameters are the same as those in other experiments. The changed parameters are only the block size and the overlapped block. When the superresolution ratio is 1 : 4, the experimental results are shown in Table 7. The obtained data is still plotted with the block size as the abscissa and PSNR values as the ordinate, as shown in Figure 11.

It can be seen from Figure 11 that the 10 × 10 training dictionary has the best superresolution reconstruction when the superresolution ratio is 1 : 4. The above experiment shows that the block size has the highest value and is related to the superresolution ratio. The larger the superresolution ratio is, the larger the block is needed. The change of the overlap block does not influence the result of the optimal block. For the MR image, the optimal block with a superresolution ratio of 1 : 2 is 5 × 5, and the optimal block with a superresolution ratio of 1 : 4 is 10 × 10.

#### 3.2.4. Number of Sampling Blocks

The experiment uses the same parameters as other experiments. The changed parameters are the sample amount of sample image blocks, and the data can be overlap extraction. The superresolution ratio is 1 : 2, and the experimental results are shown in Table 8. The data is taken as an abscissa in the image block sampling with different numbers of training dictionaries, and the image is plotted with PSNR values as the ordinate, as shown in Figure 12.

It can be seen from Figure 12 that the number of sample blocks below 10000 blocks is too small. Since the sample blocks that do not meet the requirements are removed in the algorithm, the MR images have many black or dark areas, and these gray scales are not changed much. Samples with little change in gray, all zeros, or near all zeros are rejected, which greatly reduces the number of blocks actually involved in the calculation. Therefore, as the training sample block, a training sample block with insufficient features reduces the value of PSNR when reconstructed. On the contrary, the large increase in the number of blocks does not cause a significant change in the PSNR, nor does it have a maximum value, showing a fluctuating change. All the training sample blocks participate in the training of the dictionary. Too many blocks will increase the training time, and there is no positive significance for the generation of the HD dictionary. Therefore, it is better to select 150000 sampling blocks. The following experiment with a superresolution 1 : 4 is verified.

The data in Table 9 are taken as an abscissa in the image block sampling with different numbers of training dictionaries, and the image is plotted with PSNR values as the ordinate, as shown in Figure 13. As can be seen from Figure 13, the conclusion with the superresolution ratio of 1 : 4 and is the same as that with the superresolution ratio of 1 : 2 in block selection, while the dictionary cannot be trained with a superresolution ratio of 1 : 4 when the number of blocks is 1000. There are more requirements on the number of dictionaries. Considering the reduction of dictionary training time, it is better to select 150,000 blocks.

### 3.3. Experiment Simulation of Comprehensive Parameters

The previous section analyzes several parameters that affect the superresolution effect. The values of the optimal parameters of the superresolution MR image are shown in Table 10.

The validity of the optimal parameters is verified by the experiments below. The parameters select several sets of random parameters to form a random group training dictionary, which is compared with the dictionary of optimal parameter training, as shown in Table 11. The PSNR results obtained by experiments are shown in Table 12 below.

Comparing the data in Tables 12 and 13, superresolution PSNR data in the optimal group are higher than that in the random group, no matter the superresolution ratio is 1 : 2 or 1 : 4. This shows that the parameters of the optimal group are the best parameter values.

From the experimental results can be seen, the five human body parts of the superresolution effect have obvious differences. The head and carotid artery superresolution effect is best, and ankle superresolution effect is the worst. This is mainly because each part contains different water components. More water components can produce more hydrogen protons. Under the action of magnetic field and radio frequency pulse, high-frequency information will be generated, which can better generate image edge, texture, and other details.

## 4. Conclusion

We propose a joint dictionary learning framework for superresolution of MR images, in which changes in dictionary construction parameters will cause changes in the training dictionary and thus affect the performance of superresolution reconstructed images. We have learned the optimal dictionary construction parameters through a large number of experiments and verified that the automatically learned dictionary construction parameters could effectively improve the performance of the dictionary and enhance the expression ability of the image blocks, thereby achieving better MR image superresolution effects.

## Figures and Tables

**Figure 1:** MR image superresolution architecture based on joint dictionary learning.

**Figure 2:** Image test sample. The comparison of reconstructed result with different balance parameter *λ* is shown in Table 1, where the superresolution is 1 : 2. The first column in Table 1 is the change of the balance parameter. The data in the table is the corresponding PSNR value. The results are plotted in Figure 3. (a) Head, (b) ankle, (c) carotid artery, (d) knee, and (e) neck.

**Figure 3:** PSNR curve with the balance parameter *λ* variation (superresolution ratio 1 : 4).

**Figure 4:** PSNR curve with the balance parameter *λ* variation (superresolution ratio 1 : 2).

**Figure 5:** PSNR with overlap blocks changes (superresolution ratio 1 : 2 and 1 : 4). (a) Superresolution ratio 1 : 2, (b) superresolution ratio 1 : 4.

**Figure 6:** High-resolution dictionary blocks (superresolution 1 : 2). (a) Dictionary block 3 × 3. (b) Dictionary block 6 × *c*. (c) Dictionary block 10 × 10.

**Figure 7:** Superresolution PSNR values of dictionary images constructed with different blocks (superresolution ratio 1 : 2).

**Figure 8:** High-resolution dictionary blocks (superresolution 1 : 4). (a) Dictionary block 5 × 5. (b) Dictionary block 9 × 9. (c) Dictionary block 13 × 13.

**Figure 9:** Superresolution PSNR values of dictionary images constructed with different blocks (superresolution ratio 1 : 4).

**Figure 10:** Comparison of superresolution PSNR for different blocks of a dictionary (superresolution ratio 1 : 2).

**Figure 11:** Comparison of superresolution PSNR for different blocks of a dictionary (superresolution ratio 1 : 4).

**Figure 12:** PSNR value corresponding to the training dictionary using different the number of samples (superresolution ratio 1 : 2).

**Figure 13:** PSNR value corresponding to the training dictionary using different the number of samples (superresolution ratio 1 : 4).

**Table 1:** The PSNR values of the five groups of samples with parameters *λ* variation (superresolution ratio 1 : 2).

Balance parameter *λ*	Sample 1	Sample 2	Sample 3	Sample 4	Sample 5
0.0001	32.1147	28.7875	32.0252	30.4382	30.1109
0.005	32.2643	28.9049	32.0483	30.6418	30.3621
0.01	32.2774	28.9341	32.0550	30.6463	30.3665
0.1	32.2431	28.8725	32.0357	30.5912	30.3487
0.2	32.1026	28.7828	31.9349	30.5253	30.2482
0.3	31.9502	28.6892	31.8094	30.4486	30.1392
0.4	31.7931	28.5935	31.6755	30.3667	30.0240
0.5	31.6271	28.4894	31.5267	30.2823	29.9142
0.6	31.4527	28.3712	31.3588	30.1950	29.7959
0.7	31.1624	28.1633	31.0738	30.0590	29.6033
0.8	29.1705	26.9047	29.2414	29.2739	28.1618
0.9	24.4864	23.1957	25.2566	26.5782	24.2847

**Table 2:** The PSNR values of the five groups of samples with parameters *λ* variation (superresolution ratio 1 : 4).

Balance parameter *λ*	Sample 1	Sample 2	Sample 3	Sample 4	Sample 5
0.0001	29.7593	25.2764	29.0537	26.9532	27.4701
0.005	29.8049	25.3250	29.1497	27.0742	27.5213
0.01	29.8186	25.3349	29.1571	27.0843	27.5372
0.1	29.8281	25.3454	29.1645	27.0922	27.5412
0.2	29.7391	25.2944	29.1024	27.0675	27.4779
0.3	29.6576	25.2515	29.0441	27.0382	27.4229
0.4	29.5741	25.2092	28.9856	27.0088	27.3612
0.5	29.4826	25.1631	28.9223	26.9778	27.2964
0.6	29.3861	25.1159	28.8543	26.9439	27.2285
0.7	29.2832	25.0664	28.7783	26.9074	27.1586
0.8	29.1534	25.0057	28.6830	26.8639	27.0771
0.9	28.4246	24.7130	28.1476	26.6769	26.6622

**Table 3:** The PSNR data table varies with overlap blocks.

Superresolution ratio	Overlap block	Sample 1	Sample 2	Sample 3	Sample 4	Sample 5
1 : 2	1	31.8015	28.5365	31.6296	30.3486	29.9244
1 : 2	2	31.8795	28.6155	31.7500	30.4587	30.0547
1 : 2	3	32.1207	28.8228	31.9781	30.5427	30.2708
1 : 2	4	32.2431	28.8725	32.0357	30.5912	30.3487
1 : 4	1	28.6725	24.7516	28.3602	26.6512	26.8626
1 : 4	2	29.0840	25.0284	28.6332	26.8210	27.0542
1 : 4	3	29.5786	25.2175	28.9978	27.0029	27.3708
1 : 4	4	29.8281	25.3454	29.1645	27.0922	27.5412

**Table 4:** PSNR data using different block constructed dictionaries (superresolution 1 : 2).

Dictionary blocking size	Sample 1	Sample 2	Sample 3	Sample 4	Sample 5
5 × 5	32.24	28.87	32.04	30.59	30.35
6 × 6	32.30	28.87	32.06	30.53	30.31
7 × 7	31.99	28.75	31.95	30.32	30.14
8 × 8	31.62	28.44	31.65	30.09	29.89
9 × 9	31.20	28.21	31.33	29.80	29.52
10 × 10	30.92	27.95	31.18	29.60	29.27

**Table 5:** Effects of dictionary blocks on PSNR (superresolution ratio 1 : 4).

Dictionary blocking size	Sample 1	Sample 2	Sample 3	Sample 4	Sample 5
5 × 5	29.83	25.35	29.16	27.09	27.54
6 × 6	30.00	25.49	29.38	27.22	27.72
7 × 7	30.30	25.61	29.49	27.18	27.91
8 × 8	30.40	25.71	29.72	27.23	28.02
9 × 9	30.43	25.69	29.78	27.27	28.05
10 × 10	30.75	25.75	29.94	27.32	28.11
11 × 11	30.67	25.77	29.90	27.22	28.12
12 × 12	30.53	25.71	29.82	27.19	27.93
13 × 13	30.31	25.60	29.64	27.08	27.78

**Table 6:** Comparison of superresolution PSNR for different block and overlap block training dictionaries (superresolution ratio 1 : 2).

Block size	Overlap block	Sample 1	Sample 2	Sample 3	Sample 4	Sample 5
3 × 3	2	31.30	28.21	31.22	30.26	29.70
4 × 4	3	31.96	28.70	31.73	30.54	30.19
5 × 5	4	32.24	28.87	32.04	30.59	30.35
6 × 6	5	32.29	28.90	32.07	30.55	30.32
7 × 7	6	32.11	28.83	32.03	30.40	30.26
8 × 8	7	31.90	28.71	31.93	30.26	30.08
9 × 9	8	31.71	28.60	31.80	30.10	29.93
10 × 10	9	31.43	28.42	31.65	29.95	29.70

**Table 7:** Comparison of superresolution PSNR for different block and overlap block training dictionaries (superresolution ratio 1 : 4).

Block size	Overlap block	Sample 1	Sample 2	Sample 3	Sample 4	Sample 5
3 × 3	2	29.22	25.05	28.78	26.91	27.11
4 × 4	3	29.45	25.16	28.93	26.97	27.26
5 × 5	4	29.83	25.35	29.16	27.09	27.54
6 × 6	5	30.19	25.57	29.43	27.26	27.81
7 × 7	6	30.63	25.72	29.68	27.30	28.06
8 × 8	7	30.80	25.88	29.96	27.35	28.25
9 × 9	8	30.92	25.94	30.03	27.43	28.30
10 × 10	9	31.11	25.96	30.15	27.44	28.31
11 × 11	10	30.91	25.91	30.09	27.32	28.22
12 × 12	11	30.87	25.90	30.05	27.30	28.17
13 × 13	12	30.63	25.76	29.88	27.19	27.98

**Table 8:** PSNR value corresponding to the number of sample blocks of different sampling images (superresolution ratio 1 : 2).

Number of blocks	Sample 1	Sample 2	Sample 3	Sample 4	Sample 5
1000	31.98	28.64	31.74	30.45	30.10
5000	32.15	28.79	31.94	30.52	30.23
10000	32.20	28.81	31.96	30.56	30.28
50000	32.29	28.84	31.99	30.57	30.31
100000	32.24	28.87	32.04	30.59	30.35
150000	32.31	28.91	32.04	30.60	30.37
200000	32.26	28.84	32.04	30.58	30.35
500000	32.32	28.86	32.01	30.61	30.35

**Table 9:** PSNR value corresponding to the number of sample blocks of different sampling images (superresolution ratio 1 : 4).

Number of sample image blocks	Sample 1	Sample 2	Sample 3	Sample 4	Sample 5
1000	—	—	—	—	—
5000	29.78	25.29	29.11	27.04	27.43
10000	29.75	25.30	29.15	27.09	27.48
50000	29.77	25.35	29.16	27.11	27.53
100000	29.83	25.35	29.16	27.09	27.54
150000	29.84	25.38	29.18	27.08	27.54
200000	29.81	25.36	29.17	27.09	27.51
500000	29.85	25.39	29.16	27.10	27.53

**Table 10:** MR image superresolution optimal parameters.

Super resolution ratio	Balance parameter *λ*	Overlap block	Dictionary block size	Number of sampling blocks
1 : 2	0.1	4	5 × 5	150000
1 : 4	0.1	9	10 × 10	150000

**Table 11:** List of random group parameters.

Random group	Superresolution ratio	Balance parameter *λ*	Overlap block	Dictionary block size	Number of sampling blocks
First group	1 : 2	0.1	2	4 × 4	100000
Second group	1 : 2	0.2	7	8 × 8	50000
Third group	1 : 2	0.2	4	6 × 6	10000
Forth group	1 : 2	0.3	3	7 × 7	120000
Fifth group	1 : 4	0.4	6	9 × 9	30000
Sixth group	1 : 4	0.2	4	5 × 5	80000
Seventh group	1 : 4	0.3	9	12 × 12	90000
Eighth group	1 : 4	0.1	8	10 × 10	7000

**Table 12:** PSNR data of superresolution reconstruction in random group.

Random group	Sample 1	Sample 2	Sample 3	Sample 4	Sample 5
First group	31.83	28.56	31.60	30.46	30.07
Second group	31.50	28.45	31.61	30.10	29.72
Third group	31.88	28.63	31.79	30.35	30.13
Forth group	30.78	27.85	30.87	29.74	29.17
Fifth group	30.23	25.53	29.61	27.17	27.83
Sixth group	29.80	25.34	29.14	27.07	27.50
Seventh group	30.27	25.63	29.64	27.04	27.81
Eighth group	30.66	25.81	29.85	27.28	28.06

**Table 13:** Superresolution reconstruction PSNR data in optimal group.

Optimal group	Sample 1	Sample 2	Sample 3	Sample 4	Sample 5
Super resolution ratio 1 : 2	32.31	28.91	32.04	30.60	30.37
Super resolution ratio 1 : 4	31.10	26.00	30.14	27.37	28.36

## Data Availability

We have not used specific data from other sources for the simulation of the results. The two popular MRI datasets in this paper, fast MRI Dataset and IXI Dataset, can be freely downloaded from the website https://fastmri.org/and http://www.brain-development.org/.
